# Detection of Oil Spill Using SAR Imagery Based on AlexNet Model

**DOI:** 10.1155/2021/4812979

**Published:** 2021-07-05

**Authors:** Xinzhe Wang, Jiaxu Liu, Shuai Zhang, Qiwen Deng, Zhuo Wang, Yunhao Li, Jianchao Fan

**Affiliations:** ^1^Institute of Information Science and Engineering, Dalian Polytechnic University, Dalian 116034, China; ^2^Department of Marine Remote Sensing, National Marine Environmental Monitoring Center, Dalian 116023, China; ^3^Institute of Geography Science, Liaoning Normal University, Dalian 116029, China

## Abstract

Synthetic aperture radar (SAR) plays an irreplaceable role in the monitoring of marine oil spills. However, due to the limitation of its imaging characteristics, it is difficult to use traditional image processing methods to effectively extract oil spill information from SAR images with coherent speckle noise. In this paper, the convolutional neural network AlexNet model is used to extract the oil spill information from SAR images by taking advantage of its features of local connection, weight sharing, and learning for image representation. The existing remote sensing images of the oil spills in recent years in China are used to build a dataset. These images are enhanced by translation and flip of the dataset, and so on and then sent to the established deep convolutional neural network for training. The prediction model is obtained through optimization methods such as Adam. During the prediction, the predicted image is cut into several blocks, and the error information is removed by corrosion expansion and Gaussian filtering after the image is spliced again. Experiments based on actual oil spill SAR datasets demonstrate the effectiveness of the modified AlexNet model compared with other approaches.

## 1. Introduction

Oil resources are the most important resources in the process of human industrialization. While the exploitation of marine oil enriches the oil resources, the marine oil spill caused by many factors has caused great harm to the environment. A large area of marine oil spill has caused a lot of economic losses, but at the same time, it has also caused great damage to the ecosystem. Regarding the Gulf of Mexico oil spill [1], Penglai 19-3 oil spill, and so on, those oil spill events caused damage to the local marine ecosystem and caused serious economic, ecological, and social impacts. Furthermore, the oil spill area will spread to other places with the current and wind and eventually affect a large area of the sea. Moreover, polluted marine organisms will enter the human body through the food chain, leading to a variety of diseases and even casualties [2]. Thus, the marine oil spill is one of the most serious problems of marine pollution in the world today. It should be monitored by an efficient and real-time method to extract timely information such as location and area before the oil spill is spread over a large area [3].

Because of its own characteristics, remote sensing oil spill detection technology has been a hot research field in recent years. Because aerial remote sensing, satellite remote sensing, and other remote sensing monitoring methods have the characteristics of high timeliness, high resolution, large monitoring range, not affected by regional factors, image, and graphic data are easy to process and interpret. Remote sensing monitoring provides a lot of technical support for oil spill risk inspection, oil spill pollution monitoring, early warning, emergency response, oil spill ecological damage assessment, and remediation [4].

Remote sensing images represent the differences of different ground objects through the differences of brightness value or pixel value (reflecting the spectral information of ground objects) and spatial changes (reflecting the spatial information of ground objects) [5]. In remote sensing images, the background of oil spill and seawater are different in features such as grayscale, texture, shape, and brightness. Therefore, oil spills can be identified by analyzing the feature changes of remote sensing images [6]. Early marine oil spill monitoring mainly through visual interpretation, through direct observation, or with the aid of auxiliary interpretation instrument to obtain specific target information in remote sensing images. Because the visual interpretation needs less equipment and is simple and convenient, it can obtain a lot of thematic information from remote sensing images at any time. Therefore, visual interpretation is the main method to interpret the image in the process of oil spill monitoring for a long time. However, the amount of remote sensing data is increasing year by year. Visual interpretation alone cannot meet the growing demand for monitoring. Moreover, the visual interpretation depends entirely on the experience of the interpreter, so interpretation errors are prone to occur. Therefore, computer vision is introduced into the oil spill remote sensing image monitoring. The computer or related equipment is used to simulate the biological vision, and the oil spill remote sensing image is processed to obtain the corresponding scene information. At present, an image segmentation algorithm is mainly used to extract information from oil spill remote sensing image or ENVI and another commercial remote sensing digital image processing software is used to classify sample pixels by built-in classification method [7].

The classification basis of the image segmentation algorithm is not unified, and the selection of segmentation algorithm largely depends on the shape of the image to be segmented, pixel distribution characteristics, and other factors, mainly divided into threshold segmentation, clustering segmentation, region growth, and so on.

Xu et al. applied the OTSU algorithm to oil spill monitoring [8]. Jin et al. used FCM to extract oil spill dark spots in SAR images [9]. Zou et al. used the SVM supervised classification method to complete the task of extracting oil spill information [10]. OTSU algorithm, also known as the maximum interclass variance method, was proposed by Japanese scholar OTSU in 1979. It assumes that the image to be processed only contains foreground image and background image and realizes image segmentation by calculating the threshold, which can make the maximum difference between the two types of pixels. There is also the optimal entropy threshold method proposed by Kaotur et al. and Ptile method proposed by Detcoyle et al. Clustering segmentation method is based on basic features such as grayscale pixels to divide the image according to certain rules. Then, the clustering method also developed the HCM clustering method based on a fuzzy theory proposed by RsuPini and fuzzy C-means (FCM) algorithm proposed by Dunn. The commonly used method is fuzzy C-means. The basic idea of the region growing segmentation method is to start from a group of growing points and merge the similar pixels until they cannot continue to grow.

Marine remote sensing techniques can be divided into laser fluorescence sensing, visible sensing, infrared, and microwave remote sensing [11]. The detection ability of the visible light sensor is limited due to the small contrast between the oil spill and the background. At this stage, only visible light sensor with high spatial resolution can detect oil spill effectively. However, limited by the platform, it can only be carried out in limited scenarios. Compared with laser fluorescence sensor, visible light remote sensing, infrared remote sensing, and SAR in microwave remote sensing are not limited by weather, light, and other external conditions and can monitor the target all-weather, long-term, and real-time [12]. The SAR remote sensing image with good imaging conditions has the outstanding advantages of fast, all-day, all-weather, high precision, which can penetrate the surface and vegetation to obtain the information that optical photogrammetry is difficult to obtain. The visible light remote sensing image is greatly affected by the weather, and the factors such as light, cloud, and atmospheric particles will affect the remote sensing image. Therefore, SAR has many advantages over other methods in monitoring marine oil spill and other natural disasters. In general, the most important contribution of SAR in oil spill monitoring is that it cannot be affected by rainy or cloudy weather [13]. The classical segmentation algorithms mentioned in this paper have been relatively mature and stable, but most of them have the problems of a large amount of computation and time consumption. The number of classifications (except threshold segmentation) is affected by the image itself, and it is sensitive to noise and other factors. Therefore, most of them can only be used for optical remote sensing images acquired by visible light sensors, while the classification effect of SAR images is general and unstable [14].

In recent years, deep learning has attracted extensive attention in various fields. This method mainly uses neural network to supervise the learning of samples. Deep learning has been widely used in the field of object detection. Kwan et al. used YOLO to track and classify targets [15]. As a one-stage target detection algorithm, YOLO can directly predict the whole picture. Deep learning contains many algorithms, but the most representative one is the convolutional neural network, which can be traced back to 1962, Hubel and Wiesel's research on the visual system in the cat's brain [16]. Then, the neocognitron model was proposed by Kunihiko Fukushima in 1979 and 1980. Neocognitron was a neural network with a deep structure, and it was one of the earliest deep learning algorithms. The first convolutional neural network was a time delay network proposed by Alexander Waibel in 1987 [17]. CNN is a kind of artificial neural network, and its weight-sharing network structure reduces the complexity of the network model and the number of weights. This advantage is particularly obvious when the input of the network is a multidimensional image. It can effectively learn the corresponding features from a large number of samples and extract the features better than the artificial design. Moreover, the larger the number of samples is, the better the extracted features are for classification and recognition. Meanwhile, the CNN structure has strong expansibility, and it can use a very deep number of layers. Therefore, training convolutional neural network for SAR image recognition can greatly reduce the interference caused by a lot of noise. At the same time, due to the stronger expression ability of the depth model, it has more advantages than the current mature algorithm in dealing with more complex classification problems such as remote sensing image. Convolutional neural network is used to simulate the human brain's perception of image representation. With the increasing number of iterations and the application of the optimization algorithm, the model will have better robustness. When processing SAR image, it has better performance in the face of information interference brought by more complex sea conditions. Traditional semantic segmentation algorithms are based on artificially designed features to perform segmentation, which has poor accuracy and robustness. For remote sensing images, remote sensing images have rich features. Different remote sensing images may have different characteristics of oil spills. It is difficult to find a feature that can be used to segment remote sensing images accurately [18]. However, convolutional neural network can find a feature that can segment remote sensing image accurately. Convolutional neural network is an effective method for SAR image recognition. Compared with the traditional methods, this method has better robustness and generalization ability, and the accuracy is also improved.

In SAR images, oil spill can be identified from the perspective of features such as geometry, grayscale, and texture [19]. Moreover, for different SAR remote sensing images, their characteristics are also very different. It is difficult to find suitable features that can identify oil spills. Using convolutional neural networks can avoid the process of manually searching for features. It saves the time of manually searching for suitable features and can also improve detection accuracy. Inevitably, because the imaging principle of SAR is coherent microwave imaging, this imaging principle causes the existence of coherent speckle noise in SAR remote sensing images, and the existence of coherent speckle noise makes it particularly difficult to interpret SAR images [20].

Due to the existence of coherent speckle noise, it is difficult to classify each pixel in the SAR remote sensing image like semantic segmentation. Therefore, to reduce the interference of coherent speckle noise, the larger picture is divided into many smaller pictures, and then the convolutional neural network is used to classify the cropped smaller pictures and replace the classification of each pixel in semantic segmentation by classifying the smaller pictures after cropping. In short, it uses the classification of small images to segment the original image semantically. This method not only greatly reduces the interference of speckle noise on SAR remote sensing images but also improves the detection accuracy. Because the input image is a very small image, so using a shallow network has been able to meet the requirements. The model used in this paper is the classic network model AlexNet [21]. Considering the input image is a smaller image, the model is adjusted to fit the smaller image input.

The remainder of this paper is organized as follows.  Section 2 describes the principle of convolutional neural network. The experimental methods are reported and discussed in Section 3. In Section 4, the experimental results are provided. Finally, the conclusion is given in Section 5.

## 2. Preliminary

The traditional unsupervised classification methods, such as image threshold segmentation and image edge extraction, are mainly based on the color features or texture features of the image. The extraction of image color features is to convert pixel values in digital images to corresponding values. Since color features are essentially pixel-based features, pixels in all regions of the image have corresponding contributions. As a global feature, color features are insensitive to changes in the direction and size of the image region and cannot well capture local features in the image. For texture features, this method is not like color features based on pixels but is calculated in areas containing multiple pixels. As a statistical feature, texture features usually have rotation invariance and are more resistant to noise. Texture feature is an efficient method for processing images with different thicknesses and densities. However, when the information difference between the thickness and density of the image is small, it is difficult to accurately reflect the difference between different textures perceived by human vision through texture features. When the wind wave is small, the noise is small, and the texture features of the image are relatively obvious. Images in areas with high winds and waves will appear like oil spills in texture and color. When the resolution of remote sensing images is high, this phenomenon is more obvious.

Convolutional neural network is usually composed of input layer, hidden layer, and output layer [22]. The input layer mainly performs some preprocessing operations on the picture, such as filtering and normalization. In this way, the model can be more robust.

The hidden layer usually includes the convolutional layer, the pooled layer, and the fully connected layer. The hidden layer is the key reason why CNN can extract the features of the images of the marine oil spill. Since the input image is a small image cut from the original large image, a simple convolutional neural network model can meet the requirements of the input image. For this reason, the classic AlexNet model is used. According to the size of the input image, the model is adjusted. The adjusted model includes five convolution layers: one pooling layer and three fully connected layers. After a series of convolution and pool operations, the input image is connected to the full connection layer, and two final prediction results are output, which corresponds to the score of the corresponding category.  Figure 1 shows the adjusted AlexNet model.

Finally, there is the output layer. In this part, the classification labels are output by using logical functions or normalized exponential functions, or like semantic image segmentation, the output layer directly outputs the classification results of each pixel [23].

The core of the convolutional neural network is the hidden layer. The hidden layer mainly contains three parts, the convolutional layer, the pooling layer, and the fully connected layer.

The convolution layer is the set of a series of filters, and the output of the convolution layer is called the feature map. In the process of image processing, the extraction of image features can be regarded as the solution of feature vectors. The essence of an image is a matrix composed of pixel values. Decomposition of the eigenvalues of the image is extracting the features in the image. Among them, the convolution kernel can be regarded as the eigenvector set, and the backpropagation in the hidden layer can be considered as the process of solving the eigenvector set. CNN has a better effect on Marine oil spill processing because it has certain translation invariance and rotation invariance of the image. Compared with traditional classification methods, targets can still be accurately identified when affected by unpredictable environmental factors such as thermal noise and sea waves. In the neural network, the convolution kernel is defined as the feature detector at different positions. That is, no matter where the target appears in the image, it will detect these features and output the same response. The same is true for the pooling layer. For example, the maximum pooling will return the maximum value in the field if the maximum value has been moved, but in the field, the pooling layer will still output the same maximum value. Compared with texture feature extraction, texture feature has better resistance to noise, although it usually has rotation invariance and has a good effect on processing images with great difference in thickness and density.

The pooling layer, also known as the lower sampling layer, can reduce the amount of data while retaining effective feature information. Due to the nature of the remote sensing image itself and the influence of uncertain factors such as environment, the model is prone to overfitting after processing a large amount of data. After dimensionality reduction and compression of the oil spill features that need to be extracted through the pooling layer, the overfitting will be reduced, and the fault tolerance of the model will be improved. This is especially true when extracting its features from ultrahigh resolution remote sensing images. Sampling can confuse the specific position of a feature. After a feature is found, only the relative position of this feature and other features can be needed to deal with the changes of similar objects caused by deformation and distortion.

The full connection layer is located at the last position of the whole network. From the perspective of representational learning, the full connection layer will conduct a nonlinear combination and output of the previously extracted features. That is, the full connection layer will not extract the features itself but use the extracted features at a higher stage to complete the final learning. ReLU [24] function is generally used for the excitation function of each neuron in the full connection layer. Since the ReLU function is an unsaturated nonlinear function, it can reduce the interdependence between parameters and alleviate the problem of overfitting [25]. For the problem of image classification, the output layer of the convolutional neural network generally uses the normalized exponential function to output the final classification label. Due to the small number of samples available for training oil spill images, overfitting is easy to occur. The dropout [26] operation can be introduced in the output layer to randomly delete the neurons of the neural network. Regularization and other operations can also be used to enhance the robustness of the model and reduce the phenomenon of overfitting so that the model can obtain higher accuracy in the prediction.

## 3. Oil Spill Detection Based on AlexNet

According to the principle of CNN, the extraction of the marine oil spill CNN can be roughly divided into four parts: dataset preparation, network model training, model testing, and model prediction. The specific process is shown in Figure 2.

In the preparation of the dataset, the noise generated in the SAR images in the process of imaging has the wind and waves and the ship, such as the impact of the target; scope of the different characteristics of the original data may have a very big difference, with the goal of the oil spill, features may be varied and very easy to appear in the process of training convergence, and accuracy is not high or gradient to vanish, so usually data in the input network before, need to input data standardization, namely before the convolutional neural network training data input, need in the channel or time/frequency d to normalization of data, on the image processing. The original pixel values distributed in [0, 255] are usually normalized to the range [0, 1] so that the network model has a better ability to adapt to uncontrollable factors. At the same time, due to microwave coherent imaging characters, its special imaging mechanism will bring the interference of coherent speckle noise to the image. These images with coherent speckle noise will affect the training results of the model. It is a common practice to use speckle noise reduction methods before and after prediction, which can improve the detection accuracy. Some papers in the literature have incorporated such a practice in SAR image processing [27–32]. Therefore, before the image is input to the network, the noise reduction method is used to process the image to reduce the interference of speckle noise.

In order to increase the amount of training data and improve the generalization ability and robustness of the model, the satellite remote sensing image is enhanced by inversion, translation, and rotation operations [33].

All images of datasets are processed by the cropping method. Because the predicted oil spill area and the normal sea area appear in an image at the same time, the loss of information may occur after the predicted image is restitched. Therefore, the cutting step size during cutting and splicing is smaller than the cutting size. When using the cropping method to crop a picture, if the oil spill area in the cropped picture accounts for more than 60% of the total picture, the picture will be judged as an oil spill. Otherwise, it is not judged. As shown in Figure 3, 4 *∗* 4 extraction with a step size of 2 is carried out for the region of 7 *∗* 7. The features extracted by the convolutional neural network only retain 4 *∗* 4 information after the stitching is completed. In this way, the interference between the oil spill and the image of the normal sea area is reduced, and the edge of the detection area is smoothed. At the same time, because the image size is smaller than the step size in cutting and stitching, the prediction of the following image can be used to verify the prediction result of the previous image. This method not only improves the detection accuracy but also reduces the interference of speckle noise.

In the process of the processed oil spill image entering CNN, the features are usually extracted by convolution kernel, and the features are compressed, and further dimensionality is reduced through the pooling layer [34]. These randomly initialized convolution kernels will be updated continuously through backpropagation and will approach the real solution after several iterations. The essence of this method is not to solve the whole image but to iterate out a set of feature vectors consistent with a certain distribution through the backpropagation algorithm, and this set of feature vectors infinitely approximates the conceptual feature vectors so that we can use the mathematical method of feature vectors to solve the image matrix. Therefore, CNN has the advantage that traditional feature extraction methods do not have when processing images based on remote sensing images, such as marine oil spill, whose features are difficult to separate. The convolution layer usually extracts the features of the input image through the convolution operation. The lower convolution layer extracts the relatively low-level features, such as the edges, lines, and corners of the image, while the higher the convolution layer extracts, the more advanced the features. The inner part of the convolution layer is composed of multiple convolution kernels, and each element of convolution kernels corresponds to a weight and a deviation vector. Each neuron in the convolutional layer is connected to multiple neurons in the adjacent layer above. When the convolution kernel is working, it will regularly sweep the input features and perform matrix multiplication on the input features in the receptive field and superposition of the deviation vector. The specific mathematical expression is shown as follows [35]:

(1) $$\begin{array}{c} Z^{\left(l+1\right)}\left(i,j\right)=\left[Z^{l}⊗w^{\left(l+1\right)}\right]\left(i,j\right)+b, \end{array}$$

(2) $$\begin{array}{c} \left[Z^{l}⊗w^{l+1}\right]\left(i,j\right)+b=\sum_{k=1}^{Ki}\sum_{x=1}^{J}\sum_{y=1}^{J}\left[Z_{k}^{l}\left(s_{0}i+x,s_{0}j+y\right)w_{k}^{l+1}\left(x,y\right)\right]+b. \end{array}$$

In the formula, *b* is the deviation vector, *Z*^*l*^ and *Z*^*l+1*^ represent the convolution input and output of *l + 1* layer, also known as feature map, and *L*^*l+1*^ is the size of *Z*^*l+1*^. It is assumed that the feature map has the same length and width. *Z(i, j)* corresponds to the pixels of the feature graph, where (*i*, *j*) ∈ {0,1,…, *L*_*l*+1_}, *L*_*l*+1_=(*L*_*l*_+2*p* − *f*/*sn*)+1. *K* is the number of channels of the feature graph. *f*, *s*_*0*_, and *p* are parameters of the convolution layer; they correspond to the size of the convolution kernel, the stride of the convolution, and the number of padding layers.

After the convolution layer, the output feature map is usually sent to the pooling layer for subsampling. The mathematical representation of *L*_*p*_ pooling is shown as follows [36]:

(3) $$\begin{array}{c} A_{k}^{l}\left(i,j\right)={\left[\sum_{x=1}^{f}\sum_{y=1}^{f}A_{k}^{l}{\left(s_{0}i+x,s_{0}j+y\right)}^{p}\right]}^{\left(1/p\right)}. \end{array}$$

In the formula, step size *s*_*0*_ and pixel *Z(i, j)* have the same meanings as the convolution layer, and *p* is the prespecified parameter. When *p* = 1, *L*_*p*_ pooling takes the mean value in the pooling region, which is called mean pooling. When *p* goes to infinity, *L*_*p*_ pooling takes the maximum value in the pooling region, which is called maximum pooling. The pooling layer aims to obtain spatially invariant features by reducing the resolution of the feature surface, and the pooling layer plays the role of secondary feature extraction. The pooling layer also plays the role of reducing computational complexity.

The model will be tested after training is completed every epoch. The difference between the prediction process and the final big image prediction process is that at this stage, only the small images are predicted, and the best time for model training is found by comparing the predicted results. The main purpose of this part is to measure the quality of the model.

The model prediction stage is mainly divided into 4 steps when predicting real remote sensing images. In the first step, the preprocessing stage, we will perform filtering operations on the picture to reduce the interference of coherent speckle noise in the picture. In the second step, the image is cropped according to the size of 16 *∗* 16 and the step size of 7. The third step is model prediction. The cropped images are sent with a size of 16 *∗* 16 to the trained AlexNet network for prediction. The fourth step is to generate a mask image based on the prediction result because oil spills usually exist continuously and in pieces on the sea. Therefore, a small oil spill area in the prediction result is likely to be the result of the wrong prediction. So, the oil spill area with the wrong prediction can be removed by corrosion expansion. In order to improve accuracy and reduce errors, a corrosion expansion operation is performed. This can reduce the interference to the prediction result due to the prediction error and then maps the result back to the original image to obtain the final predicted result. In this part, the adjusted AlexNet model plays the most important role, extracting features, and classification, through the classification results to determine whether it is oil spill, to generate mask image.  Figure 4 shows the detailed forecast flow chart.

In order to measure the error between the measured data and the manual calibration data, the difference between the binary image and the manually calibrated truth graph was calculated, that is, (the number of same pixels)/(the total number of pixels)  *∗* 100%, which is the accuracy. At the same time, the kappa index based on the confusion matrix is used. The kappa coefficient reflects the accuracy of classification. Under normal circumstances, the kappa coefficient range is 0-1, divided into five groups, which are very low agreement (slight) between 0.0 and 0.2 and general agreement (fair) between 0.21 and 0.40, moderate consistency between 0.41 and 0.60, substantial consistency between 0.61 and 0.80, and almost perfect between 0.81 and 1. When calculating the kappa coefficient, we need to get four data, which are the basis of the confusion matrix. They are true positive (TP), true negative (TN), false positive (FP), and false negative (FN). TP and TN mean that the predicted category of the pixel is similar to the actual category, but TP is the predicted positive category, and TN is the predicted negative category. FP and FN indicate that the predicted pixel category is not the same as the real category. The difference is that FP is the predicted positive category, while FN predicts the negative category. After obtaining the four data, *P*_*0*_ can be obtained by (4), which is the accuracy. It reflects the correct proportion of the classification. Then, *P*_*e*_ is obtained by (5), which can be called bias index. *P*_*e*_ is the product of the actual and predicted quantity/the square of the total number of samples. It reflects the balance of the results. The higher it is, the more unbalanced the confusion matrix is. And finally, kappa is obtained by combining (6). It is the evaluation index of reaction consistency standard. Also, oil spill detection aims to identify the oil spill area accurately, so the evaluation standard of recall rate shown in (7) will be used, reflecting the proportion of predicted positive samples to actual positive samples:

(4) $$\begin{array}{c} p_{0}=\frac{tp+tn}{tp+tn+fp+fn}, \end{array}$$

(5) $$\begin{array}{c} p_{e}=\frac{\left(tn+fn\right)*\left(tn+fp\right)+\left(fp+tp\right)*\left(fn+tp\right)}{{\left(tp+tn+fp+fn\right)}^{2}}, \end{array}$$

(6) $$\begin{array}{c} \text{kappa}=\frac{p_{0}-p_{e}}{1-p_{e}}. \end{array}$$

(7) $$\begin{array}{c} \text{recall}=\frac{tp}{tp+fn}. \end{array}$$

## 4. Experiments

In order to ensure the validity of this experiment, the images selected in the experiment are all SAR images with the real oil spill events.

### 4.1. Data Processing

The image is cropped by Photoshop software, and the 2109 × 2109 resolution image of some sea areas is intercepted to establish the training set. The cropped 2109 × 2109 oil spill image is cropped into multiple parts according to the method of length 16, width 16, and Step 7. In other words, the 2109 × 2109 resolution image is cropped into 300 lines  × 300 columns, and the single image size is 16 × 16 resolution image. When making the dataset, if more than 60% of the image belongs to the oil spill area, the picture is judged to be oil spill. Otherwise, it is not. During Mosaic, part of the information of a single image will be overwritten by the next adjacent image. This can improve the accuracy of detection. When making labels, if more than 60% of the part in the image belongs to the oil spill area, it is classified as the oil spill part, and the rest is classified as the nonoil spill part. After image enhancement, 90% of the labeled 16 *∗* 16 datasets (17,100 images in total) were randomly selected as training samples. A total of 1,710 images of 10% were used as test samples, and the test samples and training samples were not duplicated. Before the image is input, in order to reduce the interference caused by noise, the convolution kernel size is 3, and the mean filtering method is adopted to smooth the image. Some training samples are shown in Figure 5.

As for the model, the basic learning rate is 0.0005, and the input size is adjusted to 16 × 16 × 3. Every 50 epoch, the learning rate is adjusted once, and the adjustment magnification is 0.99, that is, adjusted to 0.99 times the previous time. The network consists of 8 layers, and the five layers are the convolution layer. After the first and second convolution layer, a maximum pooling layer is used to extract the features of the image. The last three layers are fully connected layers, which are used to classify the extracted features without updating the parameters. In order to further improve the generalization ability of the model, *L*_*2*_ regularization and dropout were used in the full connection layer during training, and the dropout parameter was set to 0.6.  Table 1 shows the detailed parameter settings of the model.

The algorithm of AlexNet is compared with OTSU, SVM, and FCM. Before the prediction, the parameters of the algorithm are set.  Table 2 shows the parameter setting of the FCM algorithm, and Table 3 shows the parameter setting of the SVM algorithm.

### 4.2. Result

The following results are from the same hardware condition. The processor is Intel(R) Core (TM) i5-10200H CPU @2.40 GHz 2.4 GHz, memory 16 GB.

There are many denoising algorithms that can deal with speckle noise, such as frost filtering and median filtering. Before image prediction, filtering the image can reduce the interference of speckle noise on the image and improve the accuracy of detection. Different denoising algorithms will produce different results. In order to select an appropriate denoising algorithm, different filtering algorithms are used for the same image, and then AlexNet is used for detection. In the detection process, only the filtering algorithm before detection is changed, and other parameters remain unchanged. Finally, recall, accuracy, and kappa coefficient are used to evaluate the results. Recall rate is the evaluation of positive samples, and oil spill detection is more concerned about the recognition effect of the oil spill area, so the use of recall rate can better compare the effect of different noise reduction algorithms. The specific results are shown in Table 4. It is not difficult to find from the table that after filtering the image, the detection accuracy is improved compared with no filtering operation, and the highest detection recall is the Lee-Sigma filter, so the Lee-Sigma filter is selected as the filtering algorithm used before image prediction.

Figure 6 shows the loss curve and precision curve.  Figure 6(a) shows the loss function and precision curve in the training process, and Figure 6(b) shows the loss function and precision curve in the verification process. It is not difficult to find that in the training process, the model's loss function is close to 0, and the accuracy is close to 1, which indicates that the model has well fitted the data of the training set. In the verification set, with the increase of epoch, the model's loss function is close to 0. The accuracy is relative to 0.96-0.97, which shows that the model has good robustness and generalization ability. The network can still achieve higher accuracy and lower loss value in few iterations at the current depth. The survey surface proves that such excellent features as CNN weight sharing greatly reduce the calculation amount during training.

In the experimental comparison results, the predicted image is obtained after corrosion expansion and smooth filtering. By macroscopic comparison between the extracted results (only after corrosion expansion treatment) and the original image, the network extraction is more accurate. Some areas that have not been accurately calibrated by human calibration can still be extracted through the network. Two criteria, accuracy and kappa coefficient, are used for image segmentation evaluation. Figures 7 and 8 are two examples of detection using different methods. They are called Sample 1 and Sample 2, respectively. Samples 1 and 2 compare the results using AlexNet, Otsu, FCM, and SVM methods, respectively. In order to maintain the fairness of the result, the same operation is performed on the predicted image before and after the prediction.

Figures 7 and 8 show the processing results of the different oil spill images by different methods. The red part is the oil spill area, and other areas are nonoil spill areas such as sea or land. Figures 7(a) and 8(a) are the original images of two different oil spill images, respectively, while Figures 7(b) and 8(b) are the results of manual annotation of these two images, respectively. Figures 7(d), 7(e), 8(d), and 8(e) show the extraction results of the same oil spill area using traditional unsupervised algorithms such as OTSU and FCM, respectively. Due to the influence of speckle noise, many speckle noises are identified as oil spill areas, and the oil spill part cannot be accurately extracted. Figures 7(f) and 8(f) show the extraction results of the SVM algorithm commonly used in supervised learning, which has high accuracy in visible light remote sensing classification. However, the algorithm is still seriously affected by noise and cannot obtain a clean oil spill area through corrosion expansion filtering. Figures 7(c) and 8(c) are the oil spill results extracted by the improved AlexNet method. It is not difficult to find that the image extraction effect is better than the other three methods. This method can not only improve the detection accuracy but also improve the detection accuracy. Because the size of clipping and stitching is smaller than the step size, the final stitching result is smoother than other methods.

After comparing the AlexNet method with OTSU, FCM, and SVM methods, the accuracy and kappa coefficient is used to evaluate the result. The specific numerical results are shown in Table 5. The most common evaluation index is accuracy, which can directly reflect the correct proportion of the results, and the calculation is straightforward. When detecting oil spills from remote sensing images, due to the uneven distribution of oil spills and nonoil spills, the oil spills only account for a small part of the whole remote sensing image. In this case, it will lead to high accuracy, which cannot well reflect the results of oil spill detection. Therefore, the kappa coefficient is added as the evaluation index. Kappa coefficient, as an index of consistency test, can better evaluate the test results.

The accuracy and kappa coefficient are used to evaluate the overall results, while in oil spill detection, the detection of oil spill area is more important than that of the nonoil spill area, so the recall rate is used to evaluate the detection results further. Recall rate reflects the proportion of predicted positive samples in actual positive samples. It only cares about positive samples, so it can better evaluate the results of oil spill detection. The specific results are shown in Table 6. It is not difficult to find that compared with other methods, the detection accuracy of AlexNet for oil spill area is much higher than the other three methods.

In addition, the time required by several detection methods is calculated. The specific time required is shown in Table 7. It is not difficult to find that the AlexNet algorithm takes the longest time. But for the oil spill detection, the detection accuracy is more important. It takes a long time to obtain higher accuracy, which is acceptable.

In order to test the generalization ability of the model, several other oil spill image input models are selected to test. These test images have different sizes and characteristics. In SAR images, the brightness of remote sensing images is different because of the different backscattering coefficients. The larger the coefficient, the brighter the image. The lower the coefficient, the darker the image. Therefore, before the image is predicted, the image's brightness to be predicted needs to be adjusted according to the image brightness standard in the training set. This can reduce the detection error caused by different image brightness. The experimental images are shown in Figure 9–13 . They are called Samples 3, 4, 5, 6, and 7, respectively.

After the picture is predicted, the results are tabulated in Table 8. It is seen that the AlexNet model has achieved good results in the picture. It has good robustness and generalization ability in detecting oil spill area.

## 5. Conclusion

By the advantage of its characterization learning ability, the CNN model achieves a high identification accuracy under the condition of small training sample size and only data enhancement and expansion capacity and extracts the oil spill areas that have not been calibrated by manual calibration. At the same time, by the advantage of its translation invariance and scaling invariance, the CNN model has good generalization ability and robustness and can still extract the oil spill area with high precision even when there is a certain difference between the two images. According to the experiment, it is feasible to use the convolutional neural network to extract the marine oil spill. YOLO model, as another small target detection scheme, can directly process the whole remote sensing imagery effectively. Thus, YOLO model can be used to detect marine oil spill in the future.

## Figures and Tables

**Figure 1:** AlexNet network model.

**Figure 2:** Flow chart of oil spill extraction.

**Figure 3:** Diagram of cutting method.

**Figure 4:** Oil spill prediction flow chart.

**Figure 5:** Partial training sample examples.

**Figure 6:** Loss and accuracy curves. (a) Train and (b) validation.

**Figure 7:** Comparison of experimental results. (a) Original SAR image. (b) The true value figures. (c) AlexNet prediction results. (d) OTSU. (e) FCM. (f) SVM.

**Figure 8:** Comparison of experimental results. (a) Original SAR image. (b) The true value figures. (c) AlexNet prediction results. (d) OTSU. (e) FCM. (f) SVM.

**Figure 9:** Comparison of experimental results. (a) Original SAR image. (b) The true value figures. (c) AlexNet prediction results.

**Figure 10:** Comparison of experimental results. (a) Original SAR image. (b) The true value figures. (c) AlexNet prediction results.

**Figure 11:** Comparison of experimental results. (a) Original SAR image. (b) The true value figures. (c) AlexNet prediction results.

**Figure 12:** Comparison of experimental results. (a) Original SAR image. (b) The true value figures. (c) AlexNet prediction results.

**Figure 13:** Comparison of experimental results. (a) Original SAR image. (b) The true value figures. (c) AlexNet prediction results.

**Table 1:** AlexNet parameters configuration.

Epoch	2500
Batch size	256
Learning rate	0.0005
Learning rate decay	0.99
Dropout	0.6
Weight decay	0.0001

**Table 2:** FCM parameters configuration.

Number of categories	2
Maximum number of iterations	50
Threshold of membership change	1e-5
Class center change threshold	1e-5

**Table 3:** SVM parameters configuration.

Kernel type	Radial basis function
Gamma in kernel function	0.333
Penalty parameter	100
Pyramid levels	0
Classification probability threshold	0

**Table 4:** Results of different filtering methods.

	Recall (%)	Accuracy (%)	Kappa
No filtering	97.88	98.52	0.78
Frost filtering	98.2	98.73	0.80
Gamma-MAP filtering	98.24	98.64	0.79
Local filtering	97.94	98.68	0.80
Mean filtering	98.26	98.58	0.79
Median filtering	98.13	98.60	0.79
Lee filtering	98.19	98.71	0.80
Lee-Sigma	98.3	98.57	0.79

**Table 5:** Test results of four methods.

Images	Overall accuracy (%)				Kappa			
	AlexNet	OTSU	FCM	SVM	AlexNet	OTSU	FCM	SVM
Sample 1	99.74	98.62	97.66	97.78	0.79	0.73	0.41	0.41
Sample 2	97.54	97.09	96.47	96.88	0.67	0.59	0.45	0.51

**Table 6:** Recall results of four methods.

Images	Recall (%)			
	AlexNet	OTSU	FCM	SVM
Sample 1	97.21	63.14	60.9	26.46
Sample 2	78.50	47.27	32.7	36.33

**Table 7:** Time of four methods.

Images	Time (s)			
	AlexNet	OTSU	FCM	SVM
Sample 1	74.32	1.63	18.36	46.16
Sample 2	70.24	1.72	21.95	43.57

**Table 8:** Experimental evaluation results.

Images	Recall (%)	Overall accuracy (%)	Kappa
Sample 3	96.32	97.73	0.70
Sample 4	99.92	93.86	0.83
Sample 5	99.76	98.91	0.73
Sample 6	96.14	96.72	0.78
Sample 7	97.24	97.93	0.83

## Data Availability

All datasets in the experiment are based on GF-3 and Radarsat‐2 SAR images, which are not freely available. These datasets can be checked and ordered from China Centre For Resources Satellite Data and Application and Canadian Space Agency.All datasets in the experiment are based on GF‐3 and Radarsat‐2 SAR images, which are not freely available. These datasets can be checked and ordered from China Centre For Resources Satellite Data and Application and Canadian Space Agency.
